# A Continuous Deep Learning System Study of Tennis Player Health Information and Professional Input

**DOI:** 10.1155/2022/8599894

**Published:** 2022-07-30

**Authors:** Lina Gong

**Affiliations:** Leisure and Sports of Xi'an I Institute Physical Education, Xi'an Physical Education University, Xi'an 710068, Shaanxi, China

## Abstract

The health status of elite tennis players and the results of tennis matches are positively proportional under normal circumstances. The physical and psychological functions of tennis players directly affect the athletic ability of tennis players. With the improvement of people's living standards, people's attention to tennis has also increased. Tennis has received increasing attention in China, and the training of tennis players has become increasingly necessary. However, China is still using the traditional means of obtaining athletes' health information to evaluate athletes' health information. This has led to imperfect research into tennis players' health information and professional input systems. This makes the understanding of the health information of athletes incomplete and profound, and it affects the athletic ability of athletes. In this paper, deep learning and a two-factor model are added to tennis players' health information and professional input, and the feasibility of a deep learning system to comprehensively improve health information input is explored. The experimental results show that the application of the convolutional neural network method in the system improves the response speed to the physical fitness state of tennis players by 5%. This adds technical support for timely understanding of tennis players' physical health information and prevents players from making mistakes on the court due to physical reasons.

## 1. Introduction

Tennis is a casual and intense sport, known as the second largest ball game in the world. In the past few years, tennis players in the country have won many championships in the international arena. The sports star effect has promoted the development of tennis in China, and people's enthusiasm for tennis has continued to grow since then. However, in professional tennis teams, there is no good solution to the problem of tennis players' health information, and players' mental and physical health information is incomplete. Many potential problems go unnoticed, and little is known about the health information of such a special group. With the emergence of these problems, the athletic level of tennis players has been affected, so many players are in poor condition on the court, and their potential has not been effectively utilized. With the increasingly widespread application of deep learning, it is necessary to build a deep learning system to apply deep learning to tennis players' health information.

The purpose of this paper is to explore the applicability of deep learning in building tennis players' health information and professional input systems. It conducts research on deep learning algorithms and analyzes the construction of continuous deep learning systems. The convolutional neural network has the advantage of extracting information about features of athletes' mental health. It iteratively calculates the information on various physical functions of athletes and obtains feedback data. This can enhance users' comprehensive understanding of tennis players' health information, effectively improve players' competitive skills, and avoid unnecessary mistakes on the court. Therefore, deep learning applications have far-reaching implications for tennis players' health information and professional input.

At present, experts' research on deep learning is becoming increasingly comprehensive and detailed. Chen Y first introduced the concept of deep learning into hyperspectral data classification. First, the applicability of stacked autoencoders was verified according to the classical classification method based on spectral information. Then a classification method based on spatial dominant information was proposed. These two features were then fused with a novel deep learning framework, from which the highest classification accuracy can be obtained. The framework is a hybrid of principal component analysis (PCA), deep learning architecture, and logistic regression. Specifically, as a deep learning architecture, stacked autoencoders aim to obtain useful high-level features. Experimental results on widely used hyperspectral data show that the classifier built in this deep learning-based framework has good performance. Furthermore, the proposed joint spectral-spatial deep neural network opens a new window for future research, demonstrating the great potential of deep learning-based methods for accurate classification of hyperspectral data [1]. Dong Y summarized recent advances in deep learning-based acoustic models and investigated the motivations and insights behind these techniques. He started by discussing models, such as recurrent neural networks and convolutional neural networks, that can effectively utilize variable-length contextual information and their various combinations with other models. He then described end-to-end optimized models, focusing on feature representations learned jointly with the rest of the system, connectionist temporal classification criteria, and attention-based sequence-to-sequence translation models. He further elaborated robustness issues in speech recognition systems and discussed acoustic model adaptation, speech enhancement and separation, and robust training strategies [2]. Wang *X* proposed an indoor positioning fingerprint system PhaseFi based on calibrated channel state information (CSI) phase information. In PhaseFi, we first extracted raw phase information from multiple antennas and multiple subcarriers of an IEEE 802.11n network interface card by accessing a modified device driver. He then used a linear transformation to extract the corrected phase information, proving that its variance is bounded. Extensive experiments are carried out in two representative indoor environments to realize and validate the proposed PhaseFi scheme. The results show that it outperforms the three benchmark schemes [3] based on CSI or received signal strength in both cases. Wu evaluated the effect of six-week respiratory muscle training on the functional performance of college tennis second-level athletes in a study of 10 healthy college tennis second-level players. They were about 18 to 25 years old and were randomly divided into two groups. Five athletes received RMT training and five other athletes received placebo training. Respiratory muscles were trained for six weeks by using the device to train inspiratory resistance loads. The different values of respiratory muscle strength and lung function were compared before and after RMT. Data analysis was performed using the Wilcoxon signed-rank test. The values of maximal expiratory pressure, physical activity, and lung function did not change significantly in this study. Conclusion: There were significant differences in maximal inspiratory pressure and diaphragm thickness after 6 weeks of respiratory muscle training. However, it is difficult to assess the effect of RMT on improving athletic performance [4]. Suna explored the effect of 21 tennis players from the Department of Sports Science who volunteered to study the effects of eight weeks of combined aerobic and anaerobic technical training on the development of athletic performance. In the study, he used flexibility, vertical long jump, standing, long jump, left-hand and right-hand grip strength, back and leg strength, anaerobic strength, 20-meter shuttle test, 5-meter and 10-meter sprint test, 1 maximum strength test, and ITN technology test. The values of flexibility, strength, 5-meter and 10-meter sprint, anaerobic capacity, 20-meter shuttle running test, and ITN technology test were compared between groups before and after training. All measurements were statistically different (*p* < 0.05). Therefore, his research found that aerobic and anaerobic combined technical training has a positive effect on biological movement, physiology, and technical characteristics [5]. Johansson F examined cumulative external workload ‘peaks' in acute/chronic workload ratios (ACWRs) for tennis training, competition, and fitness training, and whether high or low workload/age ratios are associated with back pain episodes in junior tennis players. This could affect the performance of talented young tennis players. A training program that minimizes rapid increases (peaks) in weekly training load can improve the performance and reduce back pain in junior tennis players [6]. He B found that the digital twin was an emerging smart manufacturing technology that can grasp the status of smart manufacturing systems in real time and predict system failures. Sustainable intelligent manufacturing based on digital twins has advantages in practical applications. First, he analyzed the related content of intelligent manufacturing, including intelligent manufacturing equipment, systems, and services. He then discussed the sustainability of smart manufacturing. Then, with the development of smart manufacturing based on digital twin technology, he introduced the digital twin and its applications. Finally, combined with the current situation of intelligent manufacturing, he proposed the future development direction of intelligent manufacturing [7]. These pieces of literature are very detailed for the introduction of deep learning and athlete health information, and are constructive for the research of the content of this paper.

It proposes a specific application combining deep learning, tennis player health information, and professional input, and describes the specific application process of the algorithm. It applies the two-factor model of mental health to the detection of mental health problems of tennis players and finds out the factors that affect the mental health of athletes. It feeds the tennis player's mental and physical health data into a convolutional neural network to perform computations. It explores the applicability of convolutional neural network model training in a deep learning system for tennis players' health information.

## 2. Continuous Deep Learning System Research Method for Tennis Players' Health Information and Professional Input

### 2.1. Two-Factor Model of Mental Health

#### 2.1.1. Mental Health Model of Sports Performance

A mental health model of athletic performance was proposed in 1985. This model believes that there is a relationship between athletic performance and mental health of athletes [8]. The two-factor model of mental health divides the population into four categories: completely mentally healthy, partially mentally healthy (susceptible), partially mentally disabled, and completely mentally disabled. The mental health model of athletic performance suggests that support services for athletes should not be limited to traditional preventive or therapeutic issues. Excessive psychological barriers reduce the level of the sport of athletes, which is not conducive to the healthy development of athletes. However, routine psychological screening is difficult to truly assess the fitness level of athletes. The two-factor model of mental health believes that in terms of the orientation of intervention strategies to promote mental health, on the one hand, we must continue to pursue the prevention and cure of mental disorders. At the same time, it must also pursue how to promote the psychological development of those without mental illness (low PTH) towards positive mental health.

#### 2.1.2. Athlete Psychological Intervention Model

The two-factor model of mental health believes that in the orientation of intervention strategies to promote mental health, on the one hand, we must continue to pursue the prevention and cure of mental diseases, and at the same time, we must also pursue how to promote the development of the psychology of individuals without mental diseases (low PTH) towards positive mental health. The level of the psychological level will affect the athletes' competitive performance in the arena [9]. In recent years, with the improvement of the national competition level, increasing attention has been paid to the mental health assessment of athletes. Based on the previous theoretical basis, it combines new methods, through practical experience, to conduct beneficial explorations on athletes' mental health and to carry out effective interventions. Some experts have proposed the following intervention modes [10].

#### 2.1.3. Comprehensive Model of Psychological Construction

The comprehensive model of mental construction was put forward in 1998, and its main content is to build the mental health of athletes. In response to the problems of tennis players in the game, it proposes a “a comprehensive mode of psychological construction of tennis players' game play”. As shown in Figure 1, this construction model is divided into four parts.

From the goal, the process to the result, the comprehensive model of psychological construction combines psychological training and skill training. It improves the mental health quality of tennis players and the psychological adjustment ability in actual combat [11].

#### 2.1.4. Psychological Training Hierarchical Stage Model

In 2007, a hierarchical stage model for mental training was proposed. Different from the earlier random application method, this is a multilevel and comprehensive athlete's psychological skill development model and the process of psychological intervention for athletes. The model includes two parts: psychological training and psychological counseling, as shown in Figure 2, which is a schematic diagram of the model for the hierarchical stages of psychological training.

The hierarchical stage model of psychological training gives the design process of psychological intervention strategies for athletes. It points out that sports psychology interventions should be guided by some theories. According to its specific theoretical model, it selects suitable psychological training techniques for psychological intervention. Its purpose is to focus on promoting the sports performance of athletes [12].

#### 2.1.5. Process-Level Intervention Model

It is practice-proven, psychological counseling and tennis training are combined, and psychological service goals and sports performance are consistent throughout the intervention process. It finally proposes a process-level intervention model for psychological counseling and training, as shown in Figure 3.

### 2.2. Convolutional Neural Networks

In the BP neural network, each neural node is interconnected and arranged in an orderly manner. Because of the correlation between nodes, it connects adjacent nodes with neurons, and the nodes are no longer connected, which constitutes a convolutional neural network [13]. The convolutional neural network model adopts the gradient descent method to reversely learn and correct the weight parameters in the network layer-by-layer. This minimizes the value of the cost function. It improves the accuracy of the network through frequent iterative training.

It assumes that the m-1 layer in the graph is the input layer. In BP neural network, the neuron node of this layer should be connected with all neuron nodes of the m layer. In a convolutional neural network, each neuron in the m layer is only connected to the three closest nodes to it. This greatly reduces the parameter size of the neural network architecture, as shown in Figure 4.

In the convolutional neural network, the data obtained by mental training is the input for convolution operation. It obtains the feature image of the input data and then finds the local features reflecting the rabbit from the data feature image [14]. The convolutional neural network model is also composed of input layer, hidden layer, and output layer. There are two special structural layers in the hidden layer: convolutional layer and pooling layer. A convolutional layer consists of multiple feature planes, each of which consists of neurons. Neurons on the same feature plane have the same link weights.

In the convolutional neural network, each convolution kernel of the convolution layer repeats the function of the entire receptive field and performs convolution operations on the input image. The local features of the image can be obtained from the feature map [15].

The same parameters of convolutional neural network models are shared [16], such as weight matrices and bias terms.  Figure 5 is a schematic diagram of weight sharing in a convolutional neural network. There are three neurons connected with different weight parameters. In the training process, to balance the number of parameters of the convolutional neural network, the method of gradient descent is often used to reduce the number of parameters.

Convolutional Neural Networks are actually an input-to-input process. It feeds the mental data of tennis players into a dataset and trains it through a convolutional network. The mapping relationship between each neuron is reflected, and the flow chart of convolutional neural network training is obtained, as shown in Figure 6.

The steps of the training method of convolutional neural networks are as follows:

1. Forward conduction stage
2. It first selects an input sample (*m*_*i*_, *n*_*i*_). Among them, *m*_*i*_ is used as input data, which symbolizes the input data of psychological characteristics. After convolution calculation, the corresponding output value *f*_(*m*_*i*_)_ can be obtained. During the operation, the data information goes through the operation of each convolutional layer. The calculation performed by the neural network is actually the dot product of the input value vector and the weight matrix of each layer to obtain the final output result [17].
3. Backpropagation stage
4. It comes out to define the cost function loss:

(1) $$\begin{array}{c} \text{Loss}=-\frac{1}{x}\sum_{i=1}^{x}n_{i}\text{log}f\left(m_{i}\right)+\partial \sum_{l=1}^{W}\text{sum}\left({\left\|R_{l}\right\|}^{2}\right), \end{array}$$

where *x* is the number of samples in the sample set, and W is the number of layers of the convolutional neural network.

The network parameter update needs to calculate the network parameter residual. These include the output layer residual, the residual of the convolutional layer whose next layer is the pooling layer (pooling layer), and the residual of the pooling layer whose next layer is the convolutional layer [18].

The residual calculation steps of the output layer are as follows:

For a single sample (*x*, *y*), the value of the corresponding sample cost function loss is obtained by the following formula:

(2) $$\begin{array}{c} \text{loss}=w\left(f\left(m\right),n\right)=-\sum_{c}1_{n=c}\text{log}f{\left(m\right)}_{c}=\text{log}f{\left(m\right)}_{n}. \end{array}$$

The meaning of *c* is

(3) $$\begin{array}{c} f{\left(m\right)}_{c}=k\left(n=c|m\right). \end{array}$$

It obtains the output layer residual corresponding to the loss value from the above formula:

(4) $$\begin{array}{c} \frac{\lambda }{\lambda \varepsilon^{\left(W+1\right)}}\left(-\text{log}f{\left(m\right)}_{n}\right)=-\left(e\left(n\right)-f\left(m\right)\right), \end{array}$$

where *e*(*n*) means one-hot of the sample *m* labels. Only one of the elements is 1, and the rest are 0. It yields the partial derivatives of the W layer:

(5) $$\begin{array}{c} \frac{\lambda \text{Loss}}{\lambda R_{W}}=-\frac{1}{x}\left(e\left(n\right)-f\left(m\right)*f{\left(m\right)}^{\prime }+\varepsilon R_{W}\right). \end{array}$$

It yields the partial derivative of the output layer bias. One of the matrices and one column represent a sample:

(6) $$\begin{array}{c} \frac{\lambda \text{Loss}}{\lambda o_{W}}=-\frac{1}{x}\left(e\left(n\right)-f\left(m\right)\right). \end{array}$$

It then calculates the residual of the convolutional layer of the pooling layer:

(7) $$\begin{array}{c} \infty_{j}^{t}=\text{upsample}\left(\infty^{t+1}\right)•y{\left(\ell_{j}^{t}\right)}^{\prime }. \end{array}$$

It assumes that the convolutional layer is the t-th layer, then the t+1 th layer is the pooling layer, and the residual value is (*∞*^*t*+1^). In the next layer it computes the pooling layer residuals.

It assumes that the pooling layer has *k* channels, the (*t*+1) layer has A data feature, and each channel map in the *t* layer has its own residual item. Then it gets the formula for calculating the residual of the jth channel of the *t*+1th layer:

(8) $$\begin{array}{c} \infty_{j}^{t}=\sum_{j=1}^{A}\infty^{t+1}\Theta h_{ij}. \end{array}$$

The calculation formula of the derivative of the weight and the bias value of the convolutional layer connected to the layer:

(9) $$\begin{array}{c} \frac{\lambda \text{Loss}}{\lambda h_{ij}}=m_{i}^{l}\infty^{l+1},\\ \frac{\lambda \text{Loss}}{\lambda_{k_{j}}}=\sum_{y,s}{\left(\infty^{l+1}\right)}_{y,s}. \end{array}$$

The above convolutional neural network has a total of 7 layers. The neural network converges after the number of iterations reaches 100,000. It calculates and classifies the features of data information and then outputs the required information. However, in this process, a large amount of feature data needs to be used for feature representation.

### 2.3. Recurrent Memory Network

Unlike convolutional neural networks, the main role of recurrent neural networks is to capture the characteristics of data and work with sequence data as input data [19]. It is a neural network structure with a variable input sequence and time model properties, which is extended from the former conventional neural network and linked with the recurrent neural network.  Figure 7 is a schematic diagram of the structure of the recurrent neural network. Recurrent neural networks have applications in natural language processing, such as speech recognition, language modeling, and machine translation, and are also used in various time series forecasting.

Figure 8 is a relatively original and simple structural diagram. Formally, it is given a sequence *N*=(*N*1,  *N*2,…, *Nt*), and the RNN updates its hidden state *k*_*t*_ as follows:

(10) $$\begin{array}{c} k_{t}=h\left(Q_{y_{t}}+Ph_{t-1}\right). \end{array}$$

Here, *t* ≥ 1, and g( ) is a smooth bounded function, such as a logistic function or a hyperbolic tangent function. W and U are matrices that perform the affine transformation function. The initial hidden state h0 is generally a zero vector.

When the hidden state is ht, then the probability distribution of the next element will appear in the generative expression of a recurrent neural network. It uses special symbols to represent the probability distributions of variable sequences. The probability of a sequence can be decomposed into the following formula:

(11) $$\begin{array}{c} u\left(y_{1},\ldots ,y_{T}\right)\neq u\left(y_{1}\right)u\left(y_{2}|y_{1}\right)u\left(y_{3}|y_{1},y_{2}\right)\ldots u\left(y_{T}|y_{1},\ldots ,y_{T-1}\right). \end{array}$$

The last element is a special end-of-sequence value. Then the conditional probability formula for the next sequence element is

(12) $$\begin{array}{c} u\left(y_{t}|y_{1},\ldots ,y_{t-1}\right)=h\left(h_{t}\right). \end{array}$$

In previous studies, researchers found that recurrent neural networks have long-term dependencies, and these dependencies are not captured in place. This leads to vanishing gradients and exploding gradients, which makes it more difficult to optimize gradient training networks. It is dominated by short-term dependencies not only because of changes in gradient magnitude but also because long-term impact dependencies between sequence elements are greatly weakened (exponentially decreasing relative to the sequence length). Some scholars have proposed two ways to improve the long-term dependence of recurrent neural networks. One is gradient clipping, which replaces stochastic gradient descent with a learning algorithm. It is clipped by the norm of the gradient vector in which it is clipped, or using a second-order method. If the second derivative follows the same growth pattern as the first derivative, then it may be relatively insensitive to this problem (but there is no guarantee that this will always be the case). The second is the long-short-term memory network, which consists of a more complex recurrent unit. The most representative of them is the gated cycle unit [20]. These methods can effectively improve the long-term dependence of recurrent neural networks and perform well in many tasks, such as image recognition.

### 2.4. Gradient Descent Algorithm

One of the most frequent approaches to optimization in deep learning is the gradient descent algorithm [21]. The gradient descent algorithm mainly solves the process step-by-step in an iterative manner. In this process, the stochastic gradient descent method and the batch gradient descent method are often used. To find the minimum value, the descending algorithm is used, so the gradient ascent method is used to calculate the maximum value, but a compromise is often sought according to the size of the data [22]. The theory and methods of gradient descent algorithm penetrate into many aspects, especially in military, economy, management, automatic production process, engineering design, and product optimization design.

With batch gradient descent, it uses the entire dataset (*w*, *n*) to compute the gradient, resulting in the following formula:

(13) $$\begin{array}{c} \beta =\beta -\varepsilon \cdot \nabla_{\beta }K\left(\beta ;w;n\right). \end{array}$$

When stochastic gradient descent, it uses a piece of data (*w*^(*i*)^, *n*^(*i*)^). It performs the gradient iterative calculation, resulting in the following formula:

(14) $$\begin{array}{c} \beta =\beta -\varepsilon \cdot \nabla_{\beta }K\left(\beta ;w^{\left(i\right)};n^{\left(i\right)}\right). \end{array}$$

It computes mini-batch stochastic gradient descent using a subset (*w*^(*i*; *i*+*g*)^, *n*^(*i*; *i*+*g*)^) of the full data (that is, a subset of the full data set), and the formula is

(15) $$\begin{array}{c} \beta =\beta -\varepsilon \cdot \nabla_{\beta }K\left(\beta ;w^{\left(i;i+g\right)};n^{\left(i;i+g\right)}\right). \end{array}$$

The input of the dataset is represented by w, and the label of the dataset is represented by *n*. *ε* represents the learning rate and determines the minimum moving step size. The batch size is denoted by *g*.

It can be seen from the above formula that when the calculated gradient is larger, the monthly stability of the gradient descent direction will be larger and larger. In this process, the smaller the parameter value of the update parameter, the slower the iteration speed. On the contrary, it is the opposite result [23]. In practical applications, the mini-batch gradient descent algorithm has both good stability and a more stable convergence speed. For simplicity, this article briefly introduces the mini-batch stochastic gradient descent algorithm.

In general, practical applications, there is more demand for models with large capacity. Through a series of algorithm research, the experimenter will find the best model among many algorithm models.

In practice, a model with a large capacity will be selected first, and then the capacity of the training algorithm will be controlled by some methods to find the best model in a reasonable space. The effectiveness of the algorithm depends on the number of functions in the hypothesis space and the specific form of these functions. When the input feature scale is too large, a large number of tasks will be overfitted. In deep learning, regularization methods are usually used to solve or alleviate a series of problems caused by the overfitting phenomenon. There is usually a lot of noise or random fluctuations in the data. A good fit should not be disturbed by too much noise and can effectively learn the information in the data. When a model overlearns the noise in the training data and performs poorly on new data, this phenomenon is called overfitting.

### 2.5. Regularization Methods

Regularization dominates deep learning, and only optimization can be compared to regularization [24]. One of the more interesting is the relationship between capacity and error. The error value of underfitting is too small, and overfitting is the contrast between the training error and the test error is too large, so the low-calorie model is difficult to fit for training. However, the capacity model produces overfitting during the testing process, which is not suitable for the original intention and purpose of training. Therefore, when a large number of tasks need to be solved, the regularization method in deep learning needs to be used to solve problems, such as overfitting. Among them, dropout and L2 regularization are two commonly used methods.

#### 2.5.1. Dropout

As shown in Figure 9, the schematic diagram of the neural network structure before and after applying dropout. It first randomly drops a certain percentage of neurons (and corresponding connections) from the original neural network during training. In this way, a subneural network is trained each time, preventing these neurons from overfitting the data. The traditional neural network on the left, and the neural network generated after applying dropout on the right. The red ones represent the deactivation of neurons in the neural network. During the training process, the neurons in different neural networks will be deactivated, which is a normal phenomenon in the training process. When deactivated by neurons, neurons with smaller weights are approximated, which makes the neural network training predictions tend to an average level, thereby alleviating the problem of overfitting.

#### 2.5.2. L2 Regularization

L2 regularization is to add an L2 regularization term to the model parameters after the objective function:

(16) $$\begin{array}{c} L{\left(\beta \right)}_{reg}=L\left(\beta \right)+\frac{\partial }{2N}\sum_{\beta_{i}\in w}\beta_{i}^{2}w, \end{array}$$

where *L*(*β*) is the original objective function, and *L*(*β*)_*reg*_ is the objective function after adding the L2 regular term. W is the parameter set of the model, and N is the number of model parameters. It obtains the formula for solving the derivative of the objective function with respect to the model parameters:

(17) $$\begin{array}{c} \frac{\ell L{\left(\beta \right)}_{reg}}{\beta_{i}}=\frac{\ell L\left(\beta \right)}{\beta_{i}}+\frac{\alpha }{N}\beta_{i}. \end{array}$$

It can be seen from the above formula that after adding the L2 regular term, the value of *β* becomes smaller. This shows that adding L2 to the original objective function can effectively prevent overfitting. Because when overfitting, the parameters of the fitting function are usually very large. Because the fitting function is good for each data point (including those that are abnormal or noisy), the resulting fitting function generally fluctuates greatly. In a small interval, the function value changes drastically. That is to say, when the change interval of the independent variable is small, the change of the function value is large. Then the corresponding derivative value is required to be large. This requires the coefficient to be large enough to guarantee this.

## 3. Continuous Deep Learning System Experiment of Tennis Players' Health Information and Professional Input

The health information of tennis players mainly starts from two aspects: mental health and physical health. After a scientific and in-depth analysis of the needs of tennis players, it fully reflects the overall health and trends of the players' psychological and physiological systems. This paper takes the health information detection of Chinese tennis players as the experimental object. It establishes a deep learning system for tennis players' health information from the perspective of deep learning, as shown in Figure 10 is the system function diagram.

### 3.1. Applicability of Convolutional Neural Network Model Training

The mental health data for each athlete is fed into a convolutional neural network for computation. When the system searches for the health status of an athlete, it can accurately determine the mental and physical health status of the corresponding athlete. The system cross-classifies the different state characteristics of each athlete and organizes the athlete's health information to better distinguish the characteristics of the health state.

It can be seen from Table 1 and Figure 11 that with the same weight coefficient, the orthogonal rotation begins to converge after 19 iterations. Among them, there are 11 factors with eigenvalues greater than 1, explaining 73.923% of the total variance. After the data was retested, the orthogonal rotation began to converge after 12 iterations. The iteration head starts from above 14 to below 14, and the number of iterations is 6% faster. The convergence effect is more obvious during the whole training process. Achieving a good convergence effect and increasing the number of system iterations is conducive to improving the accuracy of the detection of psychological problems in remote mobilization.

When processing the mental health information of tennis players, the amount of data is too large, which can easily lead to low work efficiency. In this paper, the regularization method in the convolutional neural network is used to detect the mental problem data of athletes. In this experiment, the following methods of analyzing fitting indicators are selected to verify the factors affecting the mental health of athletes.

It conducts sub-questionnaires on the symptoms of tennis players' mental health problems, as shown in Table 2. Among them, *χ*2/df < 2, GFI> 0.90, CFI> 0.90, and RMSEA <0.08, and the results of the positive psychological feature vector of athletes meet the system requirements. This result confirms from the side that the deep learning system of tennis players' health information based on the convolutional neural network structure is more reasonable in analyzing players' mental health problems. This also meets the criteria for evaluating the mental health of athletes.

### 3.2. Feasibility of the Two-Factor Model of Mental Health

Based on the two-factor model of psychosocial health, from the perspectives of reliability and validity, this paper explores the factors of mental problems and positive psychological characteristics of athletes. It pits 100 tennis players against subjects.  Figure 12 is the data map of common psychological problems and psychological characteristics of athletes before and after the establishment of the model.

According to the statistical results, before the model was established, tennis players had higher tendency data on the three factors of depression, hostility, and positive intelligence, which are all above 10%. After using the mental health factor model, the proportion of these factors is less than 6%. It shows that the two-factor model can effectively relieve the mental health problems of athletes under monitoring.

#### 3.2.1. Reliability Test

Reliability test refers to the test based on the reliability of the questionnaire. It is a method that uses the same experimental method to repeatedly test the results obtained on the same object to see the degree of consistency of the results. It mainly includes two parts: Cronbach's alpha coefficient and test-retest data. A simple reliability test were performed on 80 tennis players randomly selected in the system. After 15 days, it reassessed athletes' psychological problems and came up with a new sub-questionnaire for symptoms of mental health problems, whose results are shown in Table 3. In the process of reliability test, the subquestionnaire and the test of each factor are in line with the requirements of psychometrics.

#### 3.2.2. Validity Test

Validity testing refers to seeing whether it is effective to detect real things. It reflects the degree of examination content. The higher the content reflects, the higher the validity. Otherwise, it is lower. Validity tests are mainly divided into three categories: content validity, criterion validity, and construct validity. The positive psychological characteristics of athletes are one of the important indicators to evaluate the mental health of athletes. According to the validity test, 200 tennis players were selected from the system to carry out a questionnaire on positive psychological characteristics. The results are shown in Table 4. The results show that the positive mental health factors of athletes are positively correlated with the happiness index, and the psychological components of positive health reflect the positive mental characteristics of athletes. It shows that in the system test, the validity test of athletes is good.

According to Table 5, there is a moderate degree of correlation between each factor, which is lower than the correlation with the sub-questionnaire in which it is located. This shows that adding the two-factor model of mental health can make the validity test have better convergent and discriminant validity, and the factors affecting the mental health of tennis players can be detected more clearly.

From the above results, it can be seen that the indicators in the system are good and can reach the standard of psychological measurement. Therefore, the two-factor model of mental health has good applicability in this system.

### 3.3. Application of the Convolutional Neural Network in an Athlete Physiological Health Evaluation Model

The continuous deep learning research on the health information of tennis players is inseparable from various physical health checks, which can more comprehensively reflect the health information of the players. Combined with the deep learning calculation method, the classification standard of the health evaluation index of tennis players is obtained, as shown in Table 6.

According to the recurrent neural network in the convolutional neural network, it assigns a weight to the parameters of each inspection. It derives the result according to the algorithm and finally adds up the weighted scores. This completes the operation of the first-level indicator. It then obtains the health score of the secondary indicator according to the health score of the primary indicator, and then accumulates each weight. This gets the health of the primary indicator.  Table 7 is a description of the algorithm for the total score of the athlete's health. Without any restrictions, it takes the physiological health check data as individual nonlinear nodes. Convolutional neural networks can perform finite-dimensional fully connected computations. The computing power of the convolutional neural network satisfies this total score algorithm.

This algorithm is often used in speech recognition. Some experts have found through experiments that when this method is applied to the tennis players' health information detection system, the weight distribution of each indicator is scientific and reasonable for the athlete's health evaluation and the construction of a reasonable health information system. The outside world responded 5% faster to the physical fitness of tennis players. This adds technical support for timely understanding of tennis players' physical health information and prevents players from making mistakes on the court due to physical reasons.

## 4. Discussion

This paper starts from the perspective of convolutional neural networks at the deep learning level and a two-factor model of mental health. It explores the applicability of convolutional neural network model training in the deep learning system of tennis players' health information, the feasibility of the two-factor model of mental health in detecting athletes' mental health problems, the application of convolutional neural networks in athletes' physical health evaluation models, etc. The experimental results show that the deep learning system can more comprehensively and quickly reflect the physical and mental health information of athletes. It is concluded that it is reasonable and scientific to construct deep learning tennis player health information and a professional input system.

## 5. Conclusions

This paper describes the design and implementation of the algorithm for the two-factor model of mental health and the convolutional neural network. It verifies the advantages of convolutional neural networks in the calculation and arrangement of athletes' health information through experiments. It incorporates a two-factor model to gain further insight into the athlete's health information and inputs. This can effectively improve athletes' competitive skills and avoid unnecessary mistakes on the field. Therefore, deep learning is scientific and reasonable in the tennis players' health information input system. Although the applicability of deep learning is proved, the experimental data is not detailed enough, which leads to many problems in the experimental process, and it is expected that there will be better solutions in the future.

## Figures and Tables

**Figure 1:** The comprehensive mode of psychological construction of tennis players' performance.

**Figure 2:** Schematic diagram of the model for the hierarchical stages of mental training.

**Figure 3:** Tennis players' psychological counseling and a training process-level intervention model.

**Figure 4:** Schematic diagram of sparse links.

**Figure 5:** Schematic diagram of weight sharing of the convolutional neural network.

**Figure 6:** Convolutional neural network training flow chart.

**Figure 7:** Recurrent neural network structure diagram.

**Figure 8:** Left, the time series is the expanded RNN; right, RNN is expanded by the time series.

**Figure 9:** Schematic diagram of the neural network structure before and after applying dropout. (a) Standard neural network. (b) Neural network after using dropout.

**Figure 10:** Functional diagram of the deep learning system for tennis players' health information.

**Figure 11:** Gravel diagram of sample data before and after retest.

**Figure 12:** Data map of common psychological problems and psychological characteristics of athletes.

**Table 1:** KMO test for common psychological problems of athletes.

Kaiser–Meyer–Olkin with sufficient sampling		0.763
Bartlett's sphericity test	Approximate chi square	2481.734
	df	990
	Sig	0.000

**Table 2:** Athlete mental health problem symptom sub-questionnaire.

Sub-questionnaire	*χ* ^2^	df	*χ* ^2^/df	GFI	CFI	RMSEA
Symptoms of athletes' psychological problems	433.743	371	1.169	0.901	0.923	0.033
Common psychological problems of athletes	573.296	371	1.545	0.844	0.918	0.052
Positive psychological characteristics of athletes	146.741	87	1.687	0.915	0.928	0.058

**Table 3:** Reliability test table.

Factor	Cronbach's *α*coefficient	Retest coefficient
Symptoms of psychological problems	0.805	0.988^*∗∗*^
Depressed	0.856	0.954^*∗∗*^
Hostile	0.754	0.912^*∗∗*^
Anxious	0.888	0.978^*∗∗*^
Somatization	0.629	0.935^*∗∗*^

**Table 4:** The correlation between the positive psychological characteristics subquestionnaire and the well-being index of athletes.

	A	B	C	D	E	F	G	H	Population
Will quality	−0.571^*∗∗*^	−0.566^*∗∗*^	−0.483^*∗∗*^	−0.602^*∗∗*^	−0.723^*∗∗*^	−0.522^*∗∗*^	−0.368^∗^	−0.597^*∗∗*^	−0.666^*∗∗*^
Social adaptation	−0.517^*∗∗*^	−0.680^*∗∗*^	−0.322^∗^	−0.827^*∗∗*^	−0.374^∗^	−0.327^∗^	−0.166	−0.361^∗^	−0.534^*∗∗*^
Motor cognition	−0.493^*∗∗*^	−0.343^∗^	−0.326^∗^	−0.780^*∗∗*^	−0.702^*∗∗*^	−0.502^*∗∗*^	−0.381^∗^	−0.408^*∗∗*^	−0.652^*∗∗*^
Positive psychological characteristics	−0.552^*∗∗*^	−0.607^*∗∗*^	−0.482^*∗∗*^	−0.773^*∗∗*^	−0.682^*∗∗*^	−0.564^*∗∗*^	−0.345^∗^	−0.582^*∗∗*^	−0.603^*∗∗*^

**Table 5:** Correlations between various factors, factors and the total score of the subquestionnaire.

	Will quality	Social adaptation	Motor cognition
Social adaptation	0.499^*∗∗*^		
Motor cognition	0.532^*∗∗*^	0.423^*∗∗*^	
Positive psychological characteristics	0.825^*∗∗*^	0.789^*∗∗*^	0.786^*∗∗*^

**Table 6:** Classification of health evaluation indicators for tennis players.

Tennis player health information	Secondary index								
Cardiovascular system			Blood pressure				Arteriosclerosis		
Digestive and urinary system	Pancreas		Spleen	Gallbladder		Liver	Kidney		Anorectal
Respiratory system		Lung morphology			Vital capacity			FEV1.0/FVC	
Motor system		Shape			Bones			Fat	
Endocrine system		Blood			Urine			Gland	
Facial system		Oral cavity			Eye			Ear nose throat	

**Table 7:** Description of the algorithm for the total health score of athletes.

Total human health	Primary index weight	Health index grade one
J	K1	Y1
	K2	Y2
	K3	Y3
	Kn	Yn

## Data Availability

No data were used to support this study.

## References

[1] Chen Y., Lin Z., Xing Z. (2017). Deep learning-based classification of hyperspectral data[J]. *IEEE Journal of Selected Topics in Applied Earth Observations & Remote Sensing*.

[2] Dong Y., Li J. (2017). Recent progresses in deep learning based acoustic models[J]. *IEEE/CAA Journal of Automatica Sinica*.

[3] Wang X., Gao L., Mao S. (2016). CSI phase fingerprinting for indoor localization with a deep learning approach. *IEEE Internet of Things Journal*.

[4] Wu C. Y., Yang T. Y., Lo P. Y. (2017). Effects of respiratory muscle training on exercise performance in tennis players. *Medicina Dello Sport; Rivista di Fisiopatologia Dello Sport*.

[5] Suna G., Kumartaşli M. (2017). Investigating aerobic, anaerobic combine technical trainings’ effects on performance in tennis players. *Universal Journal of Educational Research*.

[6] Johansson F., Gabbett T., Svedmark P., Skillgate E. (2022). External training load and the association with back pain in competitive adolescent tennis players: results from the SMASH cohort study. *Sports Health: A Multidisciplinary Approach*.

[7] He B., Bai K. J. (2021). Digital twin-based sustainable intelligent manufacturing: a review. *Advances in Manufacturing*.

[8] Chen M., Yang J., Zhou J., Hao Y., Zhang J., Youn C. H. (2018). 5G-Smart diabetes: toward personalized diabetes diagnosis with healthcare big data clouds. *IEEE Communications Magazine*.

[9] Facs R. R. K., Sellers M. M. (2017). Invited commentary: education as a pathway to sustainable improvement. *Journal of the American College of Surgeons*.

[10] Wu J., Dong M., Ota K., Li J., Yang W. (2020). Sustainable secure management against APT attacks for intelligent embedded-enabled smart manufacturing. *IEEE Transactions on Sustainable Computing*.

[11] Li K., Zhou T., Liu B. H. (2020). Internet-based intelligent and sustainable manufacturing: developments and challenges. *International Journal of Advanced Manufacturing Technology*.

[12] Haldorai A., Chen Onn C. C., Onn M. Y., Ramu A. (2021). Intelligent pervasive computing for sustainable health-care systems. *International Journal of Pervasive Computing and Communications*.

[13] Rankin A., O’Donavon C., Madigan S. M., O’Sullivan O., Cotter P. D. (2017). Microbes in sport’ - the potential role of the gut microbiota in athlete health and performance. *British Journal of Sports Medicine*.

[14] Todd A., Eric M., David Mcduff R. (2021). Substance use and its impact on athlete health and performance[J]. *Psychiatric Clinics of North America*.

[15] Grindem H., Myklebust G. (2020). Be a champion for your athlete’s health. *Journal of Orthopaedic & Sports Physical Therapy*.

[16] Mazzeo F., Monda V., Santamaria S. (2018). Antidoping program: an important factor in the promotion and protection of the integrity of sport and athlete’s health. *The Journal of Sports Medicine and Physical Fitness*.

[17] Dai C., Lu Y. (2021). Improved biological image tracking algorithm of athlete’s cervical spine health. *Revista Brasileira de Medicina do Esporte*.

[18] Pavelko R. L., Wang T. G. (2021). Love and basketball: audience response to a professional athlete’s mental health proclamation. *Health Education Journal*.

[19] Mh A., Rh A., As B. (2020). A new method of diagnosing athlete’s anterior cruciate ligament health status using surface electromyography and deep convolutional neural network[J]. *Biocybernetics and Biomedical Engineering*.

[20] Majumder N., Poria S., Gelbukh A., Cambria E. (2017). Deep learning-based document modeling for personality detection from text. *IEEE Intelligent Systems*.

[21] Sandberg J., Barnard Y. (2018). How can deep learning advance computational modeling of sensory information processing?. *Neural and Evoultionary Computing*.

[22] June-Goo L., Sanghoon J., Young-Won C. (2017). Deep learning in medical imaging: general overview. *Korean Journal of Radiology*.

[23] Jian Y., Ni J., Yang Y. (2017). Deep learning hierarchical representations for image steganalysis. *IEEE Transactions on Information Forensics and Security*.

[24] Goh G. B., Hodas N. O., Vishnu A. (2017). Deep learning for computational chemistry. *Journal of Computational Chemistry*.

